# The Long-Term Change of Arrhythmias after Transcatheter Closure of Perimembranous Ventricular Septal Defects

**DOI:** 10.1155/2021/1625915

**Published:** 2021-06-22

**Authors:** Hongyan Zheng, Aiwen Lin, Li Wang, Yukai Xu, Zhiwei Zhang

**Affiliations:** ^1^Department of Cardiology, Cardiovascular Institute of Panyu District, Panyu Central Hospital, No. 8 Fuyudong Rd, Guangzhou City, Guangdong Province 511400, China; ^2^Department of Obstetrics and Gynecology, Panyu Central Hospital, No. 8 Fuyudong Rd, Guangzhou City, Guangdong Province 511400, China; ^3^Department of Pediatric Cardiology, Guangdong Cardiovascular Institute, Guangdong General Hospital, No. 96 Dongchuan Rd, Guangzhou City, Guangdong Province 510100, China

## Abstract

**Objectives:**

To observe and analyze the long-term change of different types of arrhythmias after transcatheter closure of perimembranous ventricular septal defect (pmVSD).

**Methods:**

We retrospectively collected the data of patients who underwent pmVSD closure in our institution from March 2002 to December 2010.

**Results:**

One hundred thirty-nine patients met the inclusion criteria, of which 265 (25.5%) had early arrhythmia. They were classified into two categories: conduction abnormality (191/1039; 18.4%) and origin abnormality (94/1039; 9.0%), including 20 patients with both types of arrhythmias. The median follow-up time was 84.5 months, and 103 patients (103/191; 53.9%) with early conduction block got permanent arrhythmias, while only three patients (3/94; 3.2%) with early anomalous origin arrhythmias still had an abnormal electrocardiogram. Serious arrhythmias (28/1039; 2.7%), including II° atrioventricular block (AVB), III° AVB, and complete left bundle branch block (CLBBB), can appear immediately in the early postoperative period (21 patients) or in the late outset (seven patients) after several months or even years (6 months to 8.3 years). Twenty patients (20/21; 95.2%) with serious arrhythmia in the early postoperative period improved after early treatment, but six patients relapsed or worsened during follow-up. At the endpoint, severe arrhythmia persisted in 13 patients, of which four patients got permanent pacemaker implanted, and one patient with recurrent CLBBB died from heart failure.

**Conclusions:**

The probability of delayed CAVB or bundle branch block after VSD closure is low but often occurs several years after surgery. Therefore, long-term ECG follow-up should last for several years or even decades. Serious arrhythmias that appear early after transcatheter pmVSD closure may impose a risk of recurrence although they have been cured already. Close attention should be paid to the changes of cardiac function in patients with CLBBB after VSD closure, and the severity of such arrhythmia should be taken seriously and reexamined.

## 1. Introduction

Ventricular septal defect (VSD) is one of the most common congenital heart malformations, accounting for 40% of all congenital heart diseases [1–3], of which the majority is perimembranous VSD (pmVSD) [4]. Currently, the treatments of pmVSD mainly include interventional occluder closure and surgical repair. Compared with the surgical repair, up to now, the interventional treatments are still controversial [5]. The initial application of Amplatzer Membranous VSD Occluder was not satisfactory in the clinical practice, which prevented the promotion and application of this technology in the United States [6]. However, kinds of VSD occluders have been widely used clinically in other countries afterwards, including China [7, 8]. In order to demonstrate the safety and performance of VSD occluders in the long run, we focused on patients with at least one-year follow-up after the procedure, since many publications only include short- or middle-term follow-up data [6, 9, 10]. Previous research has shown that the group with the AmplatzerTM Membranous and Muscular VSD occluder in child showed the highest closure rate of 93–95%, perhaps due to a better correlation between the diameter of the VSD and height of the child [11].

In China, the morbidity of complications after transcatheter pmVSD closure is decreasing in step with the increasing interventional cases [12]. Among the postoperative complications, arrhythmia happens most frequently and is the focus of most attention, especially the disturbance of conduction [11, 12]. Although it is easy to observe arrhythmias at the early postprocedures, the long-term natural process and prognosis of these operation-related arrhythmias are still uncertain.

This report described the long-term change of different types of arrhythmias in a single-center observational cohort, including 1039 consecutive patients after successful transcatheter pmVSD closure operation in Guangdong Cardiovascular Institution between 2002 and 2010 at young age, in order to find out the changing rules and risk factors of long-term arrhythmias.

## 2. Materials and Methods

### 2.1. Patient Population

Between March 2002 and December 2010, 1039 pediatric patients with pmVSD successfully underwent transcatheter device closure in Guangdong Cardiovascular Institution. Moreover, follow-up data and basic information of those patients were collected and analyzed retrospectively using medical records.

The inclusion criteria for this study included the following: (1) less than 18 years of age; (2) treatment conformed to the Chinese guideline of catheter interventional therapy for congenital heart diseases in 2004; (3) successful and safe pmVSD occluder implantation. The exclusion criteria included the following: (1) unsuccessful interventional procedure, such as the occluder not being implanted or falling off; (2) noncardiac death within one month; (3) under surgery to retrieve the occluder because of nonarrhythmias complications.

Data were collected retrospectively, including the follow-up data as well as the demographics and patients' clinical data.

### 2.2. Occluder and Procedure

Occluders used in this study included the Amplatzer VSD occlude (AGA Medical, Golden Valley, Minnesota), VSD Heart^™^ occluder (Lifetech Scientific, Shenzhen, China), and VSD Cera^™^ occluder (Lifetech Scientific, Shenzhen, China). The Amplatzer VSD occluder was eccentric, while the VSD Heart^™^ and VSD Cera^™^ occluder were eccentric, symmetry, or asymmetrical concentric. These devices have been described in detail in previous reports [13–15].

The perioperative protocol and procedure for transcatheter closure of pmVSD have been previously reported in detail [16]. All parents of the pediatric patients gave their written informed consent to the procedure.

### 2.3. Follow-Up

Clinical examination, electrocardiogram (ECG), transthoracic echocardiography (TTE), chest X-ray examination, and other examinations were performed on all subjects on the first postoperative day. The long-term outcomes of the procedure were reevaluated by ECG and TTE at 1, 3, 6, and 12 months after surgery and annually thereafter.

Postoperative arrhythmias occurring within one month were defined as early arrhythmias, while arrhythmias existing exceed one year were defined as long-term arrhythmias. Serious arrhythmias included complete atrioventricular block (CAVB), II° atrioventricular block (AVB), and complete left bundle branch block (CLBBB).

### 2.4. Statistical Analysis

All continuous variables are expressed as mean ± standard deviation (SD) or median with range as appropriate, and discrete variables are presented as frequencies and/or percentages. Statistical analysis was performed using SPSS for Windows Version 25 (IBM, Armonk, New York). Differences in categorical data were analyzed with the chi-square test. Multivariable analysis to study risk factors for the occurrence of arrhythmias was performed using multiple stepwise logistic regression analysis. The inclusion criterion was *p* < 0.05

, while removing criterion was *p* > 0.01

. All tests were two-sided. A probability value of *p* < 0.05

was considered to be statistically significant.

## 3. Results

### 3.1. Demographics and Clinical Data

One thousand thirty-nine patients were enrolled in the study. We simply divided the pmVSD into three components according to the defect location in the parasternal short-axis echo views. The inlet septum is toward between 9 and 10 o'clock, the membranous one between 10 and 11 o'clock, and the outlet one between 11 and 12 o'clock. Seventy-five patients (75/1039, 7.2%) had abnormal ECG prior to the procedure. Patients' characteristics and clinical data are described in Table 1.

### 3.2. Follow-Up

The termination of follow-up was December 2020, with the median duration time 84.5 months (1 month ∼15 years). The follow-up rate in the first month was 97.5% (1013/1039), and the first year was 84.6% (879/1039). Eight hundred thirteen patients (78.2%) completed more than five years of follow-up.

### 3.3. Early Postoperative Arrhythmias

Early postoperative arrhythmias appearing in 265 patients (25.5%) were mainly divided into two categories: (1) the conduction block abnormal arrhythmias (191/1039; 18.0%), including various degrees of atrioventricular block and types of bundle branch block; (2) the origin abnormal arrhythmias (94/1039; 9.0%), including various types of premature contractions or tachycardia. There are also 20 cases of both types of arrhythmia with conduction block and abnormal origin. Arrhythmia with the highest morbidity was right bundle branch block (RBBB), including complete or incomplete right bundle branch block, occurring in 126 patients (12.1%), followed by atrioventricular junctional tachycardia (AJT) (54/1039; 5.2%). Transient arrhythmias during procedure, minor ECG changes, such as occasion premature beats, left axis deviation, and ST segment changes were not included in this study. The incident rate of arrhythmias is described in Table 2.

Serious arrhythmias, including II° AVB, CAVB, and CLBBB, occurred in 21 patients (2.0%), of which 12 patients experienced CAVB or high-degree AVB. When severe arrhythmia, frequent premature ventricular contraction (PVC), frequent premature atrial contraction (PAC), and various types of tachycardia occurred in early postoperative period, the patients were treated with glucocorticoid (methylprednisolone 2 mg/(kg·d) or dexamethasone 0.25∼0.5 mg/(kg·d)), albumin (0.5∼1 g/(kg·d)), and myocardial nutrition medicine (creatinine phosphate (500∼1000 mg/d)). Moreover, patients with postoperative atrioventricular block would be closely observed. When the ventricular rate was too slow, a temporary pacemaker should be installed. When the medical treatment was not effect, it might even be possible to perform an operation to remove the occluder or install a permanent pacemaker with the consent of the patient's parent. Most patients with serious arrhythmias were improved after treatment, except for one with CLBBB, without the need of permanent pacemaker installation in the early postoperative period.

### 3.4. Arrhythmias during Follow-Up

At the first month after the procedure, the arrhythmias morbidity dropped to 13.5% (137/1013) compared with the early rate (265/1039, 25.5%) and further decreased to 12.7% (128/1006) in the third month and 12.5% (123/977) in the sixth month. However, at the end of follow-up, the incidence rate of arrhythmias (162/879, 18.4%) increased slightly compared with the first month (18.4% vs. 13.5%; *p*=0.005

). At the follow-up endpoint, sustained arrhythmias in 162 patients were mostly branch block (154/162, 95.1%). Long-term serious arrhythmias occurred in 14 patients, including four patients with CAVB, who underwent permanent pacemaker implantation. One patient with recurrent CLBBB had a heart failure and died at the end. The arrhythmias morbidity during the follow-up period is described in Table 2.

### 3.5. Long-Term Change of Different Types of Arrhythmias

The long-term change of different types of early arrhythmias after pmVSD closure is described as follows and in Table 3.

#### 3.5.1. CAVB or High-Degree AVB

Twelve patients, including nine with persistent CAVB, two with paroxysmal CAVB, and one with high-degree AVB, were all treated with medicines such as steroid, albumin, and myocardial nutrition immediately after AVB occurred. Of 12 patients, seven received temporary pacemaker (TP) accompanied with medicine treatment. Moreover, two patients underwent surgery to remove the occluder because of poor medical treatment. All patients were improved after treatment in the early time, without the need of permanent pacemaker. During the follow-up period, three patients experienced recurrence to CAVB or II° AVB after 19 months to 46 months after the operation. In addition, six of twelve patients got worse conduction block compared with the first month. Two patients with occluder retrieved did not get AVB recurrent or conduction block aggravation. The patients who experienced AVB recurrence or conduction block aggravation during follow-up had CAVB within five days after the closure, long-term CAVB duration (≥5 days), and large occluder size (≥8 mm). The clinical data and long-term outcomes of patients with CAVB are shown in Table 4. Except for patient no. 6 that was lost to follow-up after half a year, the rest of the patients were followed up for more than five years. Patient no. 3 experienced CAVB on the sixth day after surgery and improved after two days, but on the 14th day after the operation, CAVB was observed again and a temporary pacemaker was installed. After two days, CAVB converted to CRBBB, which continued until the end of the follow-up period.

#### 3.5.2. II° AVB

Four patients experienced a second-degree type 1 atrioventricular block in the early period. Except for one patient, which was converted to bundle branch block, all the others returned to normal ECG after medical treatment. Moreover, no recurrent or conduction block aggravation was observed during follow-up.

#### 3.5.3. I° AVB

Thirteen patients experienced I° AVB early after the procedure, including five patients who experienced accompanying bundle branch block. Until the end of the follow-up period, except for two patients who still experienced I° AVB, the rest of the patients had a normal ECG or relieved to bundle branch block, without worse conduction block.

#### 3.5.4. CLBBB

CLBBB appeared in five children in the early postoperative period, and the rest experienced CLBBB within two days after the operation. After the medical treatment, one patient still experienced CLBBB, while four patients returned to normal heart rhythm in the first month after surgery. However, at the end of the follow-up period, one patient had normal ECG, and CLBBB recurred again in three patients six months to 43 months after surgery. One child (female; 2.9 years old; 18 kg) was diagnosed with inflow tract type VSD (7.7 mm) before the operation, and a VSD Heart^™^ occluder (eccentric type, 10 mm) was inserted during the operation. The ECG changed from normal to CLBBB on the first day after the operation and returned to normal after the medical treatment. However, CLBBB recurred at the 12th month, and the echocardiogram showed that the left ventricle enlarged with unsynchronized ventricular contraction on the 20th month. The medical treatment was not effective, and the heart failure appeared to be aggravated. Cardiac resynchronization therapy (CRT) was tried, but its effect was not good. She died of cardiogenic shock within 24 hours after the CRT pacemaker implantation.

#### 3.5.5. Left Anterior Fascicular Block (LAFB) or LAFB + RBBB

Thirty-one patients had LAFB or LAFB +  RBBB. At the end of the follow-up period, 11 patients had persistent LAFB or LAFB + RBBB, and 19 experienced a relief or disappearance of conduction block. The ECG of one patient changed from double bundle branch block to normal heart rhythm in the first month but worsened to II° AVB in the fourth year and deteriorated to CAVB at the fifth year.

#### 3.5.6. RBBB

A total of 126 patients experienced complete right bundle branch block (CRBBB) or incomplete right bundle branch block (IRBBB). During the follow-up period, 41 patients had no significant changes in ECG, 68 patients experienced a relief if disappearance of abnormality, nine patients had a recurrent RBBB, and eight patients experienced worse conduction block (such as IRBBB aggravating to CRBBB or pure right bundle branch block aggravating to double bundle branch block (LAFB + RBBB)). Early CRBBB aggravated to CAVB in one patient in the third year after operation.

#### 3.5.7. Origin Abnormal Arrhythmias

Origin abnormal arrhythmias include frequent premature atrial contraction (PAC), frequent premature ventricular contraction (PVC), atrioventricular junctional tachycardia (AJT), atrial tachycardia (AT) and intermittent ventricular tachycardia (VT), and so on. Due to insufficient experience in interventional therapy in the early stage, patients with these arrhythmias in the early postoperative period were treated with glucocorticoid and other drugs. With the accumulation of interventional experience, most patients with such arrhythmias did not use glucocorticoids routinely. The long-term follow-up also indicated that most of the patients (91/94; 97%) returned to sinus rhythm, and only three patients still had intermittent ectopic tachycardia during the follow-up. In all patients, no cardiac insufficiency was found during follow-up.

#### 3.5.8. Late-Onset Arrhythmias

Of 774 patients without arrhythmia in the early postoperative period, 65 patients (65/774, 8.4%) experienced the emergence of new arrhythmias during follow-up, of which 57 experienced bundle branch block; two, I° AV; six, intermittent AJT or AT. In addition, two patients with bundle branch block in the early postoperative period developed delayed-onset CAVB in the third and fifth years of follow-up. They were treated with glucocorticoid and other drugs, but they were unable to recover and eventually received permanent pacemaker implantation. Five patients with late-onset CLBBB had normal heart rhythms in the early postoperative period, and CLBBB was dedicated six months to 8.3 years after the operation. All of them underwent cardiac echocardiography to assess the cardiac function. One of the patients had uncoordinated movement of the posterior wall of the left ventricle, but there was no clinical manifestation of heart failure and the patient is still under follow-up. The clinical data of delayed-onset severe arrhythmia after the operation is shown in Table 5.

### 3.6. Risk Factors

In the multivariate logistic regression model, the independent predictors of early postoperative arrhythmias are occluder size [*p*=0.09, *OR*: 1.087/mm (95% *CI*: 1.021∼1.157)], occluder type (asymmetrical concentric occluder) [*p*=0.01, *OR*: 1.987 (95% *CI*: 1.349∼2.926)], and the early operation date [*p*=0.038, *OR*: 1.079/year (95% *CI*: 1.004∼1.160)]. The independent predictors of serious arrhythmias during the early postoperative period include the age at operation [*p*=0.024, *OR*: 0.777/year (95% *CI*: 0.624∼0.967)] and early operation date [*p*=0.001, *OR*: 1.395/year (95% *CI*: 1.146∼1.697)]. In addition, we found that the independent predictors of long-term postoperative arrhythmias included the age at operation [*p*=0.006, *OR*: 0.921/year (95% *CI*: 0.869∼0.977)], occluder size [*p*=0.004, *OR*: 1.135/mm (95% *CI*: 1.042∼1.236)], pmVSD anatomy type (inlet septum) [*p*=0.024, *OR*: 4.092 (95% *CI*: 1.209∼13.854)], and operation date [*p* < 0.001, *OR*: 1.159/year (95% *CI*: 1.067∼1.259)] after follow-up, and the only independent predictor of long-term serious postoperative arrhythmias is the occluder type (eccentric occluder) [*p*=0.004, *OR*: 1.135 (95% *CI*: 1.042∼1.236)].

## 4. Discussion

### 4.1. Main Result

Arrhythmia, especially CAVB, is one of the most important complications after transcatheter occluder closure of pmVSD. The incident rate of arrhythmias in the early postoperative period ranges from 15.3% to 24.1% [12, 17], and CAVB rate ranges from 0.2% to 5.0% [8, 18–20]. However, most of the previous studies were limited to small series with insufficient follow-up, and most of the attention was toward the late-onset CAVB, ignoring the change in other arrhythmias. In this study, we emphasized the intermediate, long-term, and early postoperative arrhythmias in a sufficient number of patients and intended to evaluate the safety of transcatheter pmVSD closure in the long term.

The incident rate of early arrhythmias in this study was 20.5%, in agreement with previous reports. During the follow-up period, the rate of early arrhythmias was gradually decreasing, and half of the patients returned to normal. However, with the follow-up time extension, part of the patients may get recurrent or wore arrhythmias, especially those with serious arrhythmias.

Some scholars suggested that early postoperative CAVB could turn to normal or bundle branch block after a course of steroids [21, 22]. In this study, the early CAVB indeed changed to normal rhythm in an acute setting, but it could recur in long-term follow up. Nearly half of the patients experienced worse conduction block in the long term compared with the first month. It was suggested that steroids may only alleviate the myocardial edema and inflammation but will not solve the true reason for AVB occurrence, which is that the occluder had compressed the atrioventricular node. Affecting the conduction again is easy, once the proximal occluder displacement or deformation occurred. Similar cases have been reported accidentally [23]. Currently, there are few studies on late recurrence of CAVB. The recurrent time is difficult to predict, and it may be several months to several years after the surgery. In patients with late recurrent CAVB, medical treatment is ineffective, and permanent pacemaker seems the only choice [24]. It is worth mentioning that two patients in this study recovered after the occluder was removed, without conduction block aggravation or AVB recurrence. Therefore, it is debatable that patients with early CAVB should accept medical treatment or surgical occluder removal [25, 26]. Pacemaker insertion is usually recommended if there is no recovery from the AV conduction after one to two weeks [26, 27]. It remains unproven if steroids or other anti-inflammatory drugs increase the recovery rate of surgical CAVB [28, 29].

In this study, we found that patients with early CAVB occurrence time (≤5 days), long-term CAVB (≥5 days), and large occluder size (≥8 mm) experienced a high risk of conduction block aggravation or AVB recurrence. It may be suggested that we should remove the occluder from patients with early CAVB after ineffective medical treatment for five days.

This research also showed that patients with CLBBB experienced a high recurrence rate despite of early improvement after steroid treatment, and their cardiac function could decrease, accompanied with enlarging left ventricle. This might result from the damage of left ventricular systolic function and myocardial synchronize movement by CLBBB [30, 31]. In this study, one patient died of heart failure and another died of impaired cardiac function. Besides, other institutions in China also reported six patients with heart failure caused by CLBBB, of which two died [32]. The prognosis of this serious complication was terrible for the late-onset CLBBB with a poor response to steroid treatment. The cardiac resynchronization therapy proved to be effective in heart failure with CLBBB [33, 34], but not in this study. Therefore, further research is needed to confirm which treatment could be effective for patient with CLBBB and left ventricle enlarging.

Bundle branch block was a common complication with the highest incident rate both in the early and long-term follow-up. During follow-up, nearly half of the conduction block could return to normal, some of which could be worse or even deteriorate into CAVB. Some of the reported late-onset CAVB cases have been observed with different degrees of conduction block in the early postoperative period [35]. Although no cases with abnormal cardiac function causing by RBBB or LAFB had been observed, further studies are needed to clarify the long-term effects of LAFB or RBBB on cardiac function.

Origin abnormal arrhythmias, such as AJT, ectopic tachycardia, and ectopic premature beat, could almost disappear during follow-up and also had a rare recurrence. The underlying mechanism of these arrhythmias may be caused by the stimulation of the interventional device during the operation. After removing the catheters and wires in the body, the mild injury of myocardium can be improved.

Most of the patients with early rhythm in the preoperative period did not experience any change during follow-up. Some patients developed late-onset arrhythmia with an incident rate of 7.5% in this study, which is consistent with the long-term deterioration or recurrence rate of early arrhythmia (9.5%). However, this study might underestimate the incident rate of late-onset arrhythmias, because of the lower follow-up rate and shorter follow-up time compared with patients with early arrhythmias. Although most of the late-onset arrhythmias were mild ECG changes, such as RBBB, LAFB, and origin abnormality, the condition of some patients with conduction block could be worse progressively. The occurrence time could be several years or even 10 years after the operation in the study. However, now, the mechanism is uncertain. It may be relative to the inflammatory reaction or scar formation in the conduction tissue provoked by the occlude [36]. Previous research has shown that it appears to be possible that the mechanical trauma, compression, inflammation, edema, and consecutive scarring resulting in a cAVB be reduced, especially with the more flexible and softer devices [11, 37, 38].

So far, the underlying mechanism of arrhythmias after transcatheter pmVSD closure is still unclear. The risk factors may include age, weight, operation duration time, operation technique, anatomy location of the pmVSD, size of the occluder, morphological characteristics of the occluder, and so on, but the conclusions about risk factor were different in various researches [5, 12, 15, 39]. In this study, younger patients with large size occluder, asymmetrical concentric or eccentric occluder, and undergoing the operation on an early time might easily get arrhythmias. However, these risk factors have a little effect, and it is difficult to predict the probability and the exact type of arrhythmia after surgery. Some researchers even tried to use the intracardiac electrophysiology technique to predict the arrhythmias occurrence after the procedure, but the result was unsatisfying [40].

### 4.2. Clinical Implication

Considering the severity and unpredictability of the late-onset complications, proper early treatment and long-term careful follow-up of the postoperative arrhythmias are the key point of protecting patients from serious consequences.

It is unrealistic to monitor the ECG of every patient with pmVSD closure every month. Therefore, the timely detection of patients with high risk of late-onset serious arrhythmias is of great importance. In this study, we strongly suggest that patients with early serious arrhythmias should be under a careful and quite long-term follow-up, even though their ECG changed to normal after medical treatment.

Apart from the CAVB that have been reported repeatedly in previous research, the CLBBB, which was ignored formerly, should also be given the same attention. The consequence of the left ventricle enlargement caused by CLBBB is fatal and has no feasible treatment right now. Hence, it is mandatory to monitor the change of both ECG and cardiac ultrasound carefully and closely in patients with CLBBB. The echocardiographic color Doppler tissue imaging may be helpful when necessary [41].

### 4.3. Study Limitations

First, the long-term follow-up rate of patients with normal rhythm is lower than those with early arrhythmias, which raises the issue of potential bias. Second, the transient arrhythmias during interventional procedure, especially the transient AVB, were aborted in this study, because of the ignorance of operation recorder in early days. Third, it is hard to conclude the proper therapeutic protocol with statistical significance from those limited cases of serious arrhythmias. In addition, we could not summarize the rule and risk factors of the late onset arrhythmias occurring, even though we tried hard. However, the strict protocol in our institute before, during, and after the procedure made the collected data comprehensive and accurate. Lastly, the experiences of a single-center nonrandomized study may not be universally representative. Well-designed prospective cohort studies that stratify patients based on age and device type are definitely needed to establish clinical guidelines, recommending routine pmVSD transcatheter closure.

## 5. Conclusions

Percutaneous intervention pmVSD closure, which proved to be a safe and effective alternation, has been widely performed for decades. As time goes on, more and more long-term complications have been observed, such as late CAVB and heart failure caused by CLBBB. In spite of low incident rate, the late complications are not only more difficult to be discovered and cured than the early complications but also life threatening. Therefore, there is an urgent need to find out how to prevent and treat the interventional complications and establish a targeted long-term follow-up scheme.

## Figures and Tables

**Table 1:** Demographics and clinical data.

Patients (*n*)	1039
Gender (F/M) (*n* (%))	567/472 (54.6%/45.4%)
Age at operation (years)	5.2 (1.9∼17)

*Age groups (n (%))*	
＜5.0 years	505 (48.6%)
5.0∼8.0 years	271 (26.1%)
＞8.0 years	263 (25.3%)
Weight at operation (kg)	18.0 (10∼82)
VSD size (angiography) (mm)	3.6 (1.2∼16.0)

*pmVSD anatomy types (n (%))*	
Inlet septum	315 (30.3%)
Membranous septum	674 (64.9%)
Outlet septum	50 (4.8%)
Postsurgical residual VSD (*n* (%))	16 (1.5%)
Presence of aneurysm (*n* (%))	333 (32.1%)
Procedure time (min)	80.0 (30.0∼200.0).
Device size (mm)	7.0 (4∼18)

*Device corporation (n (%))*	
AGA Medical	130
Lifetech Scientific	909

*Type of device (n (%))*	
Eccentric	256 (24.6%)
Symmetric concentric	593 (57.1%)
Asymmetrical concentric	190 (18.3%)

**Table 2:** The morbidity of various types of arrhythmias during follow-up.

Arrhythmias	＜1 month (*n* = 1039)	1st month (*n* = 1013)	3rd month (*n* = 1006)	6th month (*n* = 977)	1st year (*n* = 879)	3rd year (*n* = 783)	Endpoint^1^ (*n* = 879)
CAVB or high degree AVB	12 (1.2%)	0	0	0	0	1 (0.1%)	4 (0.5%)
II° AVB	4 (0.4%)	0	0	0	0	1 (0.1%)	1 (0.1%)
I° AVB + BBB	5 (0.5%)	1 (0.1%)	1 (0.1%)	2 (0.2%)	2 (0.2%)	4 (0.5%)	0
I° AVB	8 (0.8%)	2 (0.2%)	1 (0.1%)	4 (0.4%)	2 (0.2%)	1 (0.1%)	3 (0.3%)
CLBBB	5 (0.5%)	2 (0.2%)	3 (0.3%)	3 (0.3%)	5 (0.6%)	5 (0.6%)	9 (1.0%)
LAFB + RBBB	10 (1.0%)	7 (0.7%)	7 (0.7%)	9 (0.9%)	8 (0.9%)	7 (0.9%)	11 (1.3%)
LAFB	21 (2.0%)	12 (1.2%)	12 (1.2%)	13 (1.3%)	9 (1.0%)	8 (1.0%)	10 (1.1%)
CRBBB	59 (5.7%)	53 (5.2%)	46 (4.6%)	43 (4.4%)	52 (5.9%)	56 (7.1%)	64 (7.3%)
IRBBB	67 (6.4%)	54 (5.3%)	53 (5.3%)	46 (4.7%)	52 (5.9%)	40 (5.1%)	52 (6.0%)
AJT	54 (5.2%)	1 (0.1%)	2 (0.2%)	2 (0.2%)	1 (0.1%)	2 (0.3%)	3 (0.3%)
PAC or PVC	19 (1.8%)	2 (0.2%)	1 (0.1%)	0	1 (0.1%)	2 (0.3%)	0
AT or VT	21 (2.0%)	3 (0.3%)	2 (0.2%)	1 (0.1%)	3 (0.3%)	2 (0.3%)	5 (0.6%)
Total	265^2^ (25.5%)	137 (13.5%)	128 (12.7%)	123 (12.5%)	135 (15.4%)	129 (16.5%)	162 (18.4%)

^1^The follow-up period should be more than one year, or it would not be included; ^2^20 patients with multiple types of arrhythmias were included. CAVB: complete atrioventricular block; AVB: atrioventricular block; BBB: bundle branch block; CLBBB: complete left bundle branch block; LAFB: left anterior fascicular block; RBBB: right bundle branch block; CRBBB: complete right bundle branch block; IRBBB: incomplete right bundle branch block; AJT: atrioventricular junctional tachycardia; PAC: premature atrial contraction; PVC: premature ventricular contraction; AT: atrial tachycardia; VT: ventricular tachycardia.

**Table 3:** The long-term change of different types of early arrhythmias.

Early arrhythmias	Patients, *n*	Recovered, *n* (%)	Sustained, *n* (%)	Relieved, *n* (%)	Aggravated, *n* (%)	Recurrent, *n* (%)	Median time of aggravating or recurrence (range)
CAVB or high degree AVB	12	3 (25.0%)	0	6 (50.0%)	0	3 (25.0%)	46 (19 ∼46) months
II° AVB	4	3 (75.0%)	0	1 (25.0%)	0	0	—
I° AVB + BBB	5	2 (40.0%)	0	3 (60.0%)	0	0	—
I° AVB	8	6 (75.0%)	1 (12.5%)	0	0	1 (12.5%)	6 months
CLBBB	5	1 (20.0%)	1 (20.0%)	0	0	3 (60.0%)	26 (6∼43) months
LAFB + RBBB	10	3 (30.0%)	2 (20.0%)	4 (40.0%)	1 (10.0%)	0	—
LAFB	21	12 (57.1%)	5 (23.8%)	0	0	4^1^ (19.0%)	12 (3∼69) months
CRBBB	59	20 (33.9%)	22 (37.3%)	11 (18.6%)	4 (6.8%)	2 (3.4%)	9 (3∼91) months
IRBBB	67	37 (55.2%)	19 (28.4%)	—	4 (6.0%)	7 (10.4%)	36 (1∼79) months
AJT	54	52 (96.3%)	0	—	0	2 (3.7%)	45 (3∼87) months
PAC or PVC	19	18 (94.7%)	0	—	0	1 (5.3%)	57 months
AT or VT	21	21 (100%)	0	—	0	0	—
Normal^3^	774	709 (91.6%)	—	—	65(8.4%)	—	28 (1∼101) months
Total	1039^2)^	901^2^ (86.7%)	50 (4.8%)	25 (2.4%)	74 (7.0%)	23 (2.2%)	32 (1∼101) months

^1^Two patients returned to LAFB and the other two returned and deteriorated into LAFB + RBBB. ^2^20 patients with multiple types of arrhythmias were included. ^3^No new arrhythmia appeared in the early postoperative period. CAVB: complete atrioventricular block; AVB: atrioventricular block; BBB: bundle branch block; CLBBB: complete left bundle branch block; LAFB: left anterior fascicular block; RBBB: right bundle branch block; CRBBB: complete right bundle branch block; IRBBB: incomplete right bundle branch block; AJT: atrioventricular junctional tachycardia; PAC: premature atrial contraction; PVC: premature ventricular contraction; AT: atrial tachycardia; VT: ventricular tachycardia.

**Table 4:** Clinical data of patients with CAVB or high-degree AVB.

Patient	Age (year)	Occluder type (size)	Occurrence time postoperation (day)	Therapy	AVB duration (day)	Early conversion	Long-term conversion
1	2.7	Eccentric (6 mm)	Immediately	Medicine	1	CRBBB	LAFB + IRBBB
2	6.8	Eccentric (8 mm)	4	Medicine + TP	2	CRBBB	CRBBB
3	3.8	Eccentric (8 mm)	6; 14^1^	Medicine + TP	2; 2^1^	CRBBB	CRBBB
4	4.1	Eccentric (8 mm)	4	Medicine + TP + occluder removed	4	CRBBB	CRBBB
5	3.1	Eccentric (10 mm)	5	Medicine	3	CRBBB	CLBBB
6	10.6	Symmetric (4 mm)	6	Medicine + TP	2	Normal	Normal
7	7.9	Symmetric (10 mm)	5	Medicine + TP	5	CLBBB	CAVB
8	3.3	Symmetric (10 mm)	Immediately	Medicine	7	Normal	CRBBB
9	4.3	Symmetric (10 mm)	Immediately	Medicine + occluder removed	4	IRBBB	IRBBB
10	4.6	Eccentric (8 mm)	3	Medicine + TP	9	IRBBB	CAVB
11	3.6	Eccentric (7 mm)	6	Medicine + TP	2	IRBBB	Normal
12	7.3	Symmetric (5 mm)	2	Medicine	8	Normal	II° AVB

^1^CAVB was observed again 14 days after the operation despite of relieving at the first time. TP: temporary pacemaker.

**Table 5:** Clinical data of patients with late-onset serious arrhythmias.

Patient	Age at operation (year)	Occluder type (size)	EKG at 1st day	EKG at 1st month	EKG at 1st year	EKG at last time	The time of arrhythmia (years)
1	6.17	Eccentric (6)	Normal	Normal	Normal	CLBBB	5.74
2	3.08	Eccentric (7)	Normal	Normal	Normal	CLBBB	8.33
3	6.08	Eccentric (6)	CRBBB	CRBBB	CRBBB	CAVB	3.17
4	6.33	Asymmetrical (8)	AJT	Normal	Normal	CLBBB	7.00
5	9.17	Symmetry (8)	Normal	Normal	CLBBB	CLBBB	0.50
6	3.75	Asymmetrical (6)	Normal	Normal	CLBBB	CLBBB	0.50
7	2.42	Eccentric (8)	LAFB + IRBBB	Normal	Normal	CAVB	5.00

## Data Availability

The study is a retrospective study and the research methods adopted in the study meet the requirements of scientific research ethics. The data in the article are true and valid. The data used to support the findings of this study are included within the article and also available from the corresponding author upon request.

## Additional Points

The institution at which the work was performed is Guangdong Cardiovascular Institute, Guangdong General Hospital.
